# Research and Implementation of Robot Vision Scanning Tracking Algorithm Based on Deep Learning

This article has been retracted.

**DOI:** 10.1155/2022/3330427

**Published:** 2022-07-26

**Authors:** Haifeng Guo, Wenyi Li, Na Zhou, He Sun, Zhao Han

**Affiliations:** College of Electrical and Information Engineering, Liaoning Institute of Science and Technology, Benxi, Liaoning 117004, China

## Abstract

In order to solve the difficult problem of deep learning-based robot vision tracking algorithm research and implementation, a deep learning-based target tracking algorithm and a classical tracking algorithm were proposed. It mainly uses the combination of traditional TLD algorithm and GOTURN algorithm to benefit from a large number of offline training data and updates the learner online, so that the whole system has better performance in real-time and accuracy. The results show that the performance of the TLD algorithm is poor regardless of the accuracy curve or the accuracy curve, and the performance of GOTURN-LD is significantly improved when the illumination changes. In the face of occlusion problem, the TLD algorithm shows strong robustness. Although GOTURN-LD is not very stable, its performance is better than GOTURN on the whole.

## 1. Introduction

In recent years, with the rapid development of science and technology, the application of robot technology has become the most promising field. As the computing power of graphics processor has been greatly improved, the speed of computer processing massive data has been significantly accelerated. Robot technology has been widely used in navigation and positioning, disaster rescue, unmanned driving, and other fields. In addition, China's aging population is becoming increasingly serious; so, the service robots are increasingly needed to solve the problem of labor shortages, and the basic function of the service robot is to follow the designated pedestrians and provide corresponding services at the same time [1].

The research of the robot target tracking system involves many disciplines, including computer vision, robot motion control, sensor fusion, and deep learning. The application of target tracking technology can be seen in intelligent monitoring, virtual reality, advanced human-computer interaction, motion analysis, autonomous navigation, and robot vision. For machine vision researchers, target tracking technology arouses their high research enthusiasm because it is one of the core problems in computer vision, and there are still a lot of problems to be solved [2]. Although researchers continue to try to combine the theoretical research results of mathematics, image processing, pattern recognition, artificial intelligence, machine learning, and other aspects, it is still very difficult to achieve the complete replacement of human eyes by machines.

Deep learning leads the scientific community to open the door to big data training artificial intelligence systems, leading scientists into a new era. Since 2013, deep learning has begun to show its edge in the field of target tracking and gradually shows its superiority in tracking effect [3]. Object tracking based on deep learning has two advantages. First, outperform used by the deep learning training network model is better than the traditional artificial convolutional feature representation, and as an input, it is directly used in correlation filtering or tracking framework; so, its tracking results are also better. Another advantage is it achieves end-to-end output, as long as the original image data input, the target tracking image, can be obtained.

Compared with traditional computer vision algorithms, deep learning algorithms can often provide better results because they can obtain more accurate feature expression by training a large amount of data. Therefore, deep learning technology is the mainstream solution to target tracking at present. The existing tracking algorithm based on convolutional neural network can reach the processing speed of 100 fps in video processing, which fully meets the requirements of real-time performance and has high tracking accuracy [4]. Therefore, applying deep learning to robots will be a new direction for future development of robots, and applying object tracking algorithm based on deep learning to robots will be a new direction for future development of service robots.

## 2. Literature Review

Liu et al. proposed a target tracking algorithm, which uses the Meanshift as the core, and the feature representation method of the two-digit histogram is selected by using the color and gray information of the target image to represent the target model. At the same time, combined with the motion detection module, the key information is provided for the path planning, navigation, and other high-level decisions of the autonomous mobile robot in the indoor environment [5]. Mayandi et al. built a robot sorting experimental system based on machine vision; in this system, the targets continuously enter the operation area the system controls the robot to achieve the object sorting, the system continuously and automatically obtains the image of the object through the camera, and the software analyzes the collected images, transforms the coordinates of target objects, identifies the classification information of target objects, and maintains the movement traces of sorting targets [6]. Prateek and Arya proposed a navigation method of reconnaissance robot based on visual target tracking, in which a binary robust independent element feature extraction (BRIEF) method was used to detect and describe the local invariant feature points of the visual target to be tracked, and the target localization was carried out from coarse to fine based on fast feature matching calculation. Experiments verify that this method can make the reconnaissance robot guide the target accurately in real time and accomplish the autonomous navigation task of moving to the target reliably in the complex obstacle environment [7]. Ramirez et al. proposed a mobile robot tracking system based on Kinect [8]. The skeleton tracking function of Kinect is used to identify a specific person in the depth image, and then the ranging data obtained from the Kinect sensor is used to obtain the position of the identified target in the local coordinates of the robot, and according to the law of keeping a fixed distance between human and mobile robot in depth image, a regular control law is designed to control robot movement. The experiment was done in the office corridor and showed good stability but slow response. Lvet al. proposed a DSST algorithm to study the tracking of pedestrian target by robot using monocular camera [9], which was a combination of DSST and TLD algorithm, because the DSST algorithm has no tracking failure detection mechanism, and it cannot deal with the problem of target complete occlusion. On the contrary, the TLD algorithm has tracking failure detection mechanism and can also deal with target complete occlusion. So, the advantages and disadvantages of the two algorithms are complementary, and the experimental results showed a good tracking effect. Lv et al. proposed a human visual tracking algorithm based on deep learning and probability model in order to solve the problem of service robot visual tracking for astronauts, which used deep convolutional neural network to detect the stability of the human body with various clothing and arbitrary posture, combined with the human body detection results, and the motion prediction probability model was designed to achieve accurate and continuous tracking of the designated person. The experimental results show that the proposed algorithm can track the human body stably with various clothing and arbitrary posture, and this algorithm provides an effective solution for the visual tracking of astronauts by the in-cabin following service robot in space station [10]. While the research on robot vision tracking started relatively early in foreign countries, since the 20th century, target following robots have been widely studied and applied. Creisméas et al. developed a mobile robot to locate the head position of pedestrians through skin color detection [11]. Dong et al. proposed that two panoramic stereo cameras should be vertically distributed on the top of the robot to achieve robot following [12]. Sami et al., who based on the SuperScout platform, assembled a horizontal laser scanner and then configured it on a mobile robot to sense the environment, and then go track another mobile robot [13]. In the case of low speed, the scheme can basically ensure the tracking target is not lost. Mourad et al. developed a robot which could do target tracking, and the robot could obtain the information of the tracker's back and shoulder through the camera to achieve target tracking. The powerful pattern detection and recognition system is used to solve the tracking problem in the complex background image, which makes the tracking more stable. The experimental results show that it is feasible and effective to select clothing texture and human shoulder image as the template of detection and recognition, and the tracking effect is good [14]. In the early 2000s, Segway RMP, a mobile robot tracking platform, was designed, and that robot tracking platform used LTK (Lukas-Tomasi-Kanande) feature tracking algorithm to compensate the motion of each image and calculate the difference between frames. Finally, the EM clustering algorithm was used to calculate the motion distribution of particle swarm. However, the tracking accuracy of this algorithm decreases obviously when the target moving speed increases. Li et al. developed a medical robot to assist nurses on the Kinect platform, which also had its own obstacle avoidance function and could constantly adjust the direction to avoid obstacles by judging the position of pedestrians [15] .Gao et al. proposed the tracking method of detector based on laser and RGB-D and detector that can integrate multiple associated data and Kalman filter, wanting to be implemented on a mobile robot operation system (ROS), so that in a target-dense environment, the robot can not only avoid obstacles but also intelligently detect and track specific targets [16].

## 3. Methods

### 3.1. Convolutional Layer Neural Network

The predecessor of convolutional neural network is artificial neural network, which is a unique and very important branch direction in machine learning, and a large number of studies on it contributed to the birth of convolutional neural network. Artificial neural network is a hierarchical network formed by widely connecting many simple computing units, which mimics the structure of biological neural networks and mimics the characteristics of biological neurons that can excite and inhibit, learn, and forget, providing a new solution for solving highly nonlinear and complex problems in machine learning. Firstly, the structure of artificial neural network will be briefly introduced [17].

The model of neural network can represent a very complex nonlinear function, which can express the function relation between the output signal and the input signal by the connection of multiple neurons and their hierarchical relations. Therefore, one of the characteristics of artificial neural networks is the description of nonlinear functions. The basic units of an artificial neural network are called neurons, and each neuron is shown in Figure 1.

Among them, the x1, x2,…, xn represent the input signal received by a single neuron. For each input signal, there is a weight multiplied by w1,w2,…, wn, then you take the weighted sum, and you add the offset *b* of +1 to get the sum *y*, and then *y* passes through the nonlinear and differentiable activation function *F* to obtain the output function *f* (*x*) of the weight and bias signal. The sum result *y* is abstracted by mathematical formula, as shown in Formula (1):

(1) $$\begin{array}{c} y=f\left(\overset{n}{\underset{i=1}{\sum }}w_{i}x_{i}+b\right). \end{array}$$

If there is no activation function to transform the sum *y*, then the single neuron model can only deal with the antecedent problem, if activation function is added, nonlinear transformation will be realized, so that neurons can deal with complex problems. The above activation function *f* usually uses sigmoid function and ReLU function. Here, we use the sigmoid function as an example, sigmoid function expression, which maps the weighted sum to (0, 1), and derivative, *σ*′(*z*) = *σ*(*z*)(1 − *σ*(*z*)), has good mathematical properties [18], as shown in Formula (2):

(2) $$\begin{array}{c} \sigma \left(z\right)=\frac{1}{1+e^{-z}}. \end{array}$$

Then, the final output result expression of the single neuron model is shown in Formula (3):

(3) $$\begin{array}{c} y=f_{w,b}\left(x\right)=\frac{1}{1+\exp\left(-\sum_{i}w_{i}x_{i}-b\right)}. \end{array}$$

Multiple simple neurons are connected in parallel and combined hierarchically to form a neural network model, as shown in Figure 2. God network is divided into three parts: input layer, hidden layer, and output layer. Layer L1 is the input layer, layer L2 and layer Ln-1 are the hidden layer, and layer Ln is the output layer. The number of hidden layers and the number of neurons in each layer are set artificially, while the number of nodes in input and output layers is fixed and related to tasks. Each layer of neurons is fully connected to the next layer, but there is no connection between the neurons of this layer; in the figure, except the node with the value of+1 represents the bias term *b*, each of the remaining connecting lines represents a weight *w*, and the arrow direction indicates the direction of data flow during forward network operation.

In Figure 2, the neural network has *N* layers, and suppose the activation functions are sigmoid functions, called *σ*_*l*_(*l* = 2, ⋯, *n*), *w*_*ij*_^*l*^ is used to represent the connection weight value of the *j*-th neuron at layer l-1 and the *i*-th neuron at layer l, and weights and bias items will be constantly modified to minimize the error of the model during training, if *u*_*i*_^*l*^ and *y*_*i*_^*l*^ are used to represent the input and output values of the *i*-th neuron in layer l, respectively; so, the relationship of each value in the forward operation of the network will be as follows:

(4) $$\begin{array}{c} \left\{\begin{array}{c} y_{i}^{\prime }=\sigma \left(u_{i}^{\prime }\right)\\ u_{i}^{\prime }=\underset{j}{\sum }w_{ij}^{l-1}y_{j}^{l-1} \end{array}\right.\;\;l=1,2,\cdots ,n \end{array}$$

The advantages of the convolutional neural network model lie in three core aspects. The first is local perception, also known as local connection. Each neuron only connects with small local regions in the previous layer. By taking advantage of the characteristics of strong correlation between regions with close distances in the image and weak distance, then local information is integrated at a higher level to obtain global information, thus to reduce the number of parameter training. The second is shared weight, which on the basis of local connection to further reduce the number of parameters. Since some features in the image will appear repeatedly in other positions, the same weight can be used to carry out convolution calculation for different regions of the image, independent of the local position of the image. And the last is multiconvolution kernels, and the weights and offsets are called the convolution kernel or filter [19]. A convolution kernel represents a feature. In order to obtain different feature sets, the convolution layer has multiple convolution kernels to generate different features.

### 3.2. GOTURN-LD Algorithm Design

#### 3.2.1. Advantages and Disadvantages of TLD Algorithm

Tracking-Learning-Detection (TLD) is a new tracking framework proposed in 2012, which can effectively decompose complex tracking tasks into three parts. The tracker retrieves two frames of data, and then the forward trajectory of the target feature point from the previous frame to the target feature point in the current frame is calculated by using pyramid LK optical flow method and next calculate the reverse trajectory, and finally, based on the results, the target position information of the current frame is predicted. The detector is responsible for collecting target characteristics and background information and marks the target as a positive sample and the background as a negative sample, and then the scanned samples are sent to the learner through three cascade classifiers to distinguish positive and negative samples. The learner updates the target model by adjusting parameters, mainly according to the results of the detector, so as to prevent the occurrence of wrong sample values in the future. TLD developed a new learning method, P-N learning, which estimates the sample error by a pair of P-N experts [20]. The learning process is modeled as a discrete dynamic system, and the learning module is improved in the dynamic adjustment. After extensive quantitative evaluation analysis, it shows a significant improvement over the traditional tracking algorithm. The whole structure is shown in Figure 3.

The advantage of the TLD algorithm lies in the tracking failure detection mechanism, which enables TLD to complete the long-term tracking task, but most algorithms lack this mechanism; so, it can only be tracked for a short time. Since the algorithm has a global detection module, that is, detection capability, when the target deformation is too large or is completely blocked, leading to tracking failure, the algorithm will detect the target in each subsequent frame of the image, and the tracking will resume as soon as the target is detected[21]. The disadvantage of the TLD algorithm lies in the tracking module. The tracking algorithm used by the module is the pyramid LK optical flow tracking method. The tracking algorithm is greatly affected by lighting, and it is easy to lead to the tracking failure of the LK algorithm when the target moves fast or the target has nonrigid deformation. Therefore, the TLD algorithm is suitable for tracking small targets with stable illumination, significant illumination, no background, and no violent movement.

#### 3.2.2. Advantages and Disadvantages of GOTURN Algorithm

The advantage of the GOTURN algorithm lies in its fast tracking speed, up to 100 fps, which is better than most algorithms based on deep learning, which generates a Generic Object Tracking during the training phase. In the test phase, no tuning is required, tracing is performed directly, computation is reduced, and the speed is increased. At the same time, the influence of illumination on target tracking is reduced by using convolutional neural network to extract features.

The disadvantage of the GOTURN algorithm is that the effect is poor with occlusion, since the algorithm uses logistic regression, and the assumption of this regression method is that the target moves slowly, and there is no occlusion. The algorithm is suitable for short time tracking and has no tracking failure detection mechanism. If the target is occluded and tracking drift occurs, it cannot be retrieved due to the lack of detection module. After the above analysis, the advantages and disadvantages of TLD algorithm and GOTURN algorithm are summarized, and GOTURN-LD considering the combination of the advantages of the two algorithms, an improved tracking algorithm GOTURN-LD is proposed based on the redesigned tracking module and detection module [22].

#### 3.2.3. GOTURN-LD Algorithm Design

The improvement of the GOTURN-LD algorithm is mainly based on TLD framework, using track-detection framework. The improvement not only overcomes the defect of TLD algorithm tracking module but also changes GOTURN, which can only track for a short time, into a long time tracking. In addition, the detection module of GOTURN-LD is improved, which reduces time-consuming calculation and affect the sample size of target model; so, it not only speeds up the retrieval speed after occlusion or loss but also improves the detection accuracy and makes the algorithm more reliable [23].

The tracking module of the TLD algorithm uses the pyramid LK optical flow tracking method, which is a fast tracking algorithm with the image as the input and the target box as the output, and GOTURN is also an end-to-end algorithm. Therefore, the tracking module of TLD algorithm can be replaced by GOTURN algorithm, while other modules remain unchanged, so that GOTURN algorithm can be combined with TLD algorithm to form a new GOTURN-LD algorithm.

In the tracking module, since the input and output of GOTURN and TLD algorithms are consistent, therefore, the tracking algorithm is regarded as a black box, and the GOTURN algorithm can be directly used to replace the LK optical flow tracking method. However, the TLD trace module has a trace failure detection mechanism; so again, a failure detection method suitable for the GOTURN algorithm needs to be designed [24]. We know that the GOTURN trace will receive two inputs; after clipping, the similarity of the two images will be calculated. If the similarity is too small, it means the tracing fails; so, the detection module is required to scan the image. So the target model needs to be updated, and the trace module needs to be reinitialized. Referring to the TLD tracking module, the error square and *D* as measuring standards are chosen, and the calculation formula is shown in Formula (5):

(5) $$\begin{array}{c} D\left(i,j\right)=\underset{\left(i,j\right)\in w}{\sum }{\left(I_{1}\left(i,j\right)-I_{2}\left(i,j\right)\right)}^{2}. \end{array}$$

Here, *i* and *j* represent pixel points, I1 and I2 represent the corresponding gray values of the clipping graph of the previous frame and the current frame, respectively. After the test, it is found that when *D* is greater than 0.7, the error is large, and the similarity is small, which is judged as tracking failure.

And then we use the strategy of hierarchical grouping, in which way we calculate the similarity and next merge these subregions are which are used as candidate images. The similarity is expressed as formula (6):

(6) $$\begin{array}{c} s\left(r_{i},r_{j}\right)=a_{1}s_{\text{color}}\left(r_{i},r_{j}\right)+a_{2}s_{\text{size}}\left(r_{i},r_{j}\right) \end{array}$$

Colors represent the color similarity, and the expression is shown in formula (7):

(7) $$\begin{array}{c} s_{\text{color}}\left(r_{i},r_{j}\right)=\overset{n}{\underset{k=1}{\sum }}\min\left(c_{i}^{k},c_{j}^{k}\right). \end{array}$$

Size represents the scale similarity, and im represents the merged region, as shown in Formula (8):

(8) $$\begin{array}{c} S_{\text{size}}\left(r_{i},r_{j}\right)=1-\frac{\text{size}\left(r_{i}\right)+\text{size}\left(r_{j}\right)}{\text{size}\left(im\right)}. \end{array}$$

An image block *P* and a target model *M* are given arbitrarily and then use the correlation similarity index to determine the target area, and the correlation similarity ranges from 0 to 1. The larger the value, the more similar it is, and the more likely it is to be the target region. The calculation formula of correlation similarity is shown in Formula (9):

(9) $$\begin{array}{c} S^{r}=\frac{S^{+}}{S^{+}+S^{-}}. \end{array}$$

The definition of image similarity is shown in Formula (10), and NCC is the normalized crossrelation number.

(10) $$\begin{array}{c} S\left(p_{i},p_{j}\right)=0.5\left(\text{NCC}\left(p_{i},p_{j}\right)+1\right). \end{array}$$

With the target model, the image blocks output in the previous step can be detected and classified. The final image block is output by judging whether its correlation similarity is greater than the given threshold value. The image block that passes through the three cascaded classifiers is the final output of the detection module, that is, the positive sample [25].

## 4. Experimental Results and Discussion

In the actual verification, the effect is not good because of the delay of network video transmission. So, a laptop instead of a server to deal with computing problems is chosen, a camera instead of a webcam to deal with video streaming is chosen, and through USB to connect the camera to the laptop is chosen. The tracking system framework of the test is shown in Figure 4.

In order to evaluate the performance of the algorithm in more detail, OTB50, a traditional data set in the field of target tracking, was chosen to carry out specific experiments. OTB50 provides video sequences with 11 target variation challenges and 51 video sequences with real target locations. There are usually three quantitative evaluation indexes of OTB50, which are OPE, TRE, and SRE. OPE refers to the tracking evaluation by initializing the tracker through the artificially calibrated initialization box of the first frame; TRE refers to the evaluation of the robustness of a tracking algorithm over time; SRE refers to the evaluation of the robustness of tracking algorithms from space. For each metric, there are precision plot and success plot plots to show performance.

Since only illumination and occlusion are considered, six representative video sequences such as David and woman are selected to test and compare the performance of TLD, GOTURN, and GOTURN-LD algorithms. We choose SRE index to analyze the algorithm from the success rate and accuracy rate, respectively, see Figures 5 and 6.

When the illumination changes, the performance of the TLD algorithm is poor, whether the accuracy curve or the accuracy curve, and the performance of GOTURN-LD is significantly improved. When faced with occlusion problem, The TLD algorithm shows strong robustness. However, GOTURN-LD is not very stable, and its overall performance is better than GOTURN. These two points also verify the performance of the proposed improved algorithm, and it does combine the advantages of the two algorithms. The overall performance is good. The real-time analysis of the algorithm usually uses the tracking speed as the evaluation index, and the tracking speed is expressed by frame/s. Similarly, six videos such as David and woman in OTB50 were selected as test sequences. After testing and comparing the tracking speeds of GOTURN-LD, TLD, and GOTURN algorithms, the results are shown in Figure 7.

According to the results, the GOTURN-LD algorithm failed to show the high speed of the GOTURN algorithm because of the detection mechanism, but compared with the TLD algorithm, it has some advantages. In general, it can basically meet the real-time requirements.

## 5. Results

The difficult problem of research and implementation of the robot vision tracking algorithm based on deep learning are solved. By analyzing the target tracking algorithm based on deep learning and classical tracking algorithm, their advantages and disadvantages are analyzed, and some suggestions for improvement are put forward. The traditional TLD algorithm combined with the GOTURN algorithm is mainly adopted, benefits from a large amount of offline training data are gained, and the learner online is updated, so that the whole system has a better performance in real-time and accuracy. As for the improved algorithm, the robot vision tracking system based on deep learning is mainly composed of two parts: a server that integrates high-performance GPU and a multifunctional intelligent robot with depth camera. The experimental process of the designed system in the test environment is as follows: first, the server takes visual information from the network and processes it with core deep learning algorithms by using monocular cameras to collect visual information to obtain information about the location of the target to be tracked; then, the location information is sent to the intelligent robot. The intelligent robot completes the machine movement according to the obtained position information to achieve the effect of target tracking. And it turns out, for single target tracking, the system designed in this paper has a good performance on the problems of illumination change, target occlusion, and reappearance after disappearance.

## Figures and Tables

**Figure 1:** Diagram of a single neuron model.

**Figure 2:** Simple neural network.

**Figure 3:** TLD algorithm framework.

**Figure 4:** Actual development environment diagram.

**Figure 5:** SRE success rate curves for illumination and occlusion problems.

**Figure 6:** SRE accuracy curves for illumination and occlusion problems.

**Figure 7:** Tracking speed comparison (frames/s) of GOTURN-LD, TLD, and GOTURN.

## Data Availability

The data used to support the findings of this study are available from the corresponding author upon request.
